RETRACTED

# Distinct Molecular Subtypes of Diffuse Large B Cell Lymphoma Patients Treated with Rituximab-CHOP Are Associated with Different Clinical Outcomes and Molecular Mechanisms

**DOI:** 10.1155/2021/5514726

**Published:** 2021-06-19

**Authors:** Haifeng Yu, Shuailing Peng, Shuiyun Han, Xi Chen, Qinghua Lyu, Tao Lei

**Affiliations:** ^1^Department of Lymphatic Medical Oncology, The Cancer Hospital of the University of Chinese Academy of Sciences (Zhejiang Cancer Hospital), Institute of Basic Medicine and Cancer (IBMC), Chinese Academy of Sciences, Hangzhou, 310022 Zhejiang, China; ^2^Cancer Institute (Key Laboratory of Cancer Prevention & Intervention, National Ministry of Education, Provincial Key Laboratory of Molecular Biology in Medical Sciences), The Second Affiliated Hospital Zhejiang University School of Medicine, Hangzhou, 310009 Zhejiang, China

## Abstract

**Objective:**

Our purpose was to characterize distinct molecular subtypes of diffuse large B cell lymphoma (DLBCL) patients treated with rituximab-CHOP (R-CHOP).

**Methods:**

Two gene expression datasets of R-CHOP-treated DLBCL patients were downloaded from GSE10846 (*n* = 233, training set) and GSE31312 (*n* = 470, validation set) datasets. Cluster analysis was presented via the ConsensusClusterPlus package in R. Using the limma package, differential expression analysis was utilized to identify feature genes. Kaplan-Meier survival analysis was presented to compare the differences in the prognosis between distinct molecular subtypes. Correlation between molecular subtypes and clinical features was analyzed. Based on the sets of highly expressed genes, biological functions were explored by gene set enrichment analysis (GSEA). Several feature genes were validated in the molecular subtypes via qRT-PCR and western blot.

**Results:**

DLBCL samples were clustered into two molecular subtypes. Samples in subtype I displayed poorer overall survival time in the training set (*p* < 0.0001). Consistently, patients in subtype I had shorter overall survival (*p* = 0.0041) and progression-free survival time (*p* < 0.0001) than those in subtype II. Older age, higher stage, and higher international prognostic index (IPI) were found in subtype I. In subtype I, T cell activation, lymphocyte activation, and immune response were distinctly enriched, while cell adhesion, migration, and motility were significantly enriched in subtype II. T cell exhaustion-related genes including TIM3 (*p* < 0.001), PD-L1 (*p* < 0.0001), LAG3 (*p* < 0.0001), CD160 (*p* < 0.001), and CD244 (*p* < 0.001) were significantly highly expressed in subtype I than subtype II.

**Conclusion:**

Two molecular subtypes were constructed in DLBCL, which were characterized by different clinical outcomes and molecular mechanisms. Our findings may offer a novel insight into risk stratification and prognosis prediction for DLBCL patients.

RETRACTED

## 1. Introduction

Diffuse large B cell lymphoma (DLBCL) is the most common aggressive non-Hodgkin's lymphoma globally [1]. According to different cell origins, DLBCL is divided into three subtypes including germinal center B cell-like (GCB; 41%) and activated B cell-like (ABC; 35%) subtypes and others based on gene expression profile, which has become the standard method of prognosis in clinical practice [2]. Nevertheless, its prognostic effectiveness of this classification has not been uniformly proven due to the heterogeneity of classification structures [3]. The international prognostic index (IPI) is an effective clinical tool for predicting risk stratification and prognosis. However, it cannot guide personalized therapy [4]. The rituximab, cyclophosphamide, doxorubicin, and prednisone (R-CHOP) therapy is currently proven to be one of the most effective treatment regimen for most DLBCL subtypes. However, approximately 40% of patients will experience fatal recurrence or progression [5]. The 5-year overall survival rate of patients receiving first-line treatment is 60-70% [6]. Through the first-line treatment of R-CHOP, most patients can be completely relieved. However, due to obscure reasons, some individuals in remission will develop relapse [7]. Hence, it is of importance to develop a novel prognostic stratification tool to accurately predict the prognosis of patients treated with R-CHOP and identify those who will experience immunosuppressive chemotherapy resistance.

Next-generation sequencing technology offers novel insights for individualized therapy of DLBCL patients. Moreover, some promising targets have been detected for the prevention and treatment of relapsed/refractory DLBCL [8]. For instance, coexpression of CD5 and CD43 may predict a poor prognosis of DLBCL patients [9]. A high NEAT1_1 level is positively correlated with stage, IPI, extranodal involvement, drug response, and poor prognosis [10]. Furthermore, LAMP1 expression is in relationship with IPI, overall survival, and progression-free survival for DLBCL [11]. Despite these biomarkers predicting the clinical outcomes of DLBCL, none of them have been translated into clinical practice. Thus, this study is aimed at screening and validating potential biomarkers for predicting survival outcomes of DLBCL patients and serving as therapeutic targets.

There is high heterogeneity in immune cells surrounding malignant B cells, which is related to the prognosis of DLBCL patients [12–14]. Chronic inflammation in DLBCL can suppress the differentiation and proliferation of T cells, caused by the continuous expression of inhibitory receptors, such as LAG3 and TIM3 [15]. By the suppression of the immune response, tumor cells are protected from immune surveillance [15]. It has been strikingly highlighted that the heterogeneity of DLBCL is reflected in molecular subtypes at the transcriptional level, which can provide insights into pathogenesis and candidate therapeutic targets for DLBCL [16]. Thus, it is of importance to characterize molecular subtypes of R-CHOP-treated DLBCL patients. Based on gene expression profiles of DLBCL, we aimed to characterize molecular subtypes with distinct prognoses and clinical features, which might improve the treatment strategy of DLBCL and prolong high-risk patients' survival time.

RETRACTED

## 2. Materials and Methods

### 2.1. Data Collection and Preprocessing

From the Gene Expression Omnibus (GEO) repository (https://www.ncbi.nlm.nih.gov/gds/), we searched the gene expression profiles of DLBCL samples according to the following criteria: (1) patients were treated with R-CHOP, (2) patients had complete follow-up information, and (3) the number of patients was over 200. As a result, GSE10846 and GSE31312 datasets were included in this study. The GSE10846 dataset including 233 DLBCL patients treated with R-CHOP based on the GPL570 [HG-U133_Plus_2] Affymetrix Human Genome U133 Plus 2.0 Array platform was used as the training set [17, 18]. The GSE31312 dataset including 470 DLBCL patients on the platform of GPL570 [HG-U133_Plus_2] Affymetrix Human Genome U133 Plus 2.0 Array was utilized as the validation set. When a gene corresponded to multiple probes, we took the average value as the expression value of the gene. Clinical information including age, stage, sex, IPI, overall survival time, and disease-free survival time was also extracted from the two datasets. Among them, the IPI scoring standard is based on the patient's age, general condition score, clinical stage, involvement of extranodal sites, and lactate dehydrogenase.

### 2.2. Consensus Cluster Analysis

Consensus cluster analysis was performed to determine the optimal clustering number (*k*) by the ConsensusClusterPlus package in R [19]. The stability of the cluster was evaluated through resampling-based methods.

### 2.3. Differential Expression Analysis

Differential expression analysis was presented between the two molecular subtypes on raw data or Microarray Analysis (limma) package in R [20]. Genes with a false discovery rate (FDR) < 0.05 were set as feature genes. On the basis of these feature genes, the samples in the validation set were used for cluster analysis via the nearest template prediction (NTP) algorithm [21].

RETRACTED

### 2.4. Kaplan-Meier Survival Analysis

Kaplan-Meier overall and progression-free survival was presented for patients between the two molecular subtypes via Survival package in R, which was assessed by the log-rank test. The definition of overall survival refers to the time from the beginning of randomization to the death of a patient from any cause. Progression-free survival is defined as the time from diagnosis to any cause leading to progression, recurrence, or death. Multivariate Cox regression analysis was presented to assess whether the molecular subtypes could independently predict overall and progression-free survival time following adjusting gene expression profile classification.

### 2.5. Gene Set Enrichment Analysis (GSEA)

Gene Ontology (GO) biological process enrichment analysis was separately presented on the basis of two sets of highly expressed genes in the two molecular subtypes using the GSEA software (http://software.broadinstitute.org/gsea/index.jsp) [22, 23]. The number of permutations was set as 1000. Adjusted *p* value < 0.05 was set as the threshold value.

### 2.6. Correlation Analysis

We further analyzed the relationships between the molecular subtypes and other clinical factors including age, stage, sex, and IPI. The differences between the two subtypes were assessed via the Wilcoxon rank-sum test.

### 2.7. Patient Samples

Totally, 30 DLBCL patients and matched 30 healthy individuals were recruited in The Cancer Hospital of the University of Chinese Academy of Sciences between 2019 and 2020 in this study. All patients were diagnosed by experienced pathologists. Formalin-fixed paraffin-embedded (FFPE) biopsy specimens were used for qRT-PCR and western blots. Each patient signed an informed consent form. This research project gained the approval of The Cancer Hospital of The University of Chinese Academy of Sciences ethics committee (2019-037).

### 2.8. Quantitative Real-Time PCR (qRT-PCR)

After the tissue was lysed by TRIzol (15596-018; Invitrogen, Carlsbad, California, USA), the sample was transferred to a 1.5 ml EP tube. 200 *μ*l chloroform (100006818; Sinopharm Chemical Reagent Co., Ltd, Shanghai, China) was added to the EP tube and left at room temperature for 5 min. After 12000 rpm centrifugation for 15 min at 4°C, the upper aqueous phase was transferred to a new 1.5 ml EP tube; 400 *μ*l isopropanol (A507048; Sangon Biotech, Shanghai) was added and allowed to stand at room temperature for 10 min. Following centrifugation at 12000 rpm for 10 min at 4°C, the supernatant was discarded. A spectrophotometer (752; Shanghai Sunny Heng Scientific Instrument Co., Ltd.) was used to determine RNA concentration. The total RNA was reverse transcribed into cDNA via the RNA cDNA first strand synthesis kit (AT341; TransGen Biotech, Beijing, China). Fluorescence quantitative PCR detection was presented by the ABI StepOnePlus type fluorescence quantitative PCR instrument. GAPDH was used as an internal control.  Table 1 lists the information of primers.

RETRACTED

### 2.9. Western Blot

The tissue samples were lysed in RIPA lysis buffer (P0013B; Beyotime, Beijing, China) at 4°C for 30 min. The protein concentration was determined with the BCA kit (P0010; Beyotime). The absorbance at OD568 was measured with a microplate reader (EPOCH2; BioTek, Vermont, USA). The sample was separated by SDS-PAGE gel and transferred to a PVDF membrane. The PVDF membrane was sealed with TBST blocking solution containing 5% skimmed milk powder at room temperature for 30 min. The membrane was incubated with the primary antibodies against CD244 (1 : 1000; ab196745; Abcam, USA), TIM3 (1 : 1000; ab185703), CD160 (1/200; ab202845), LAG3 (1 : 1000; ab237718), and GAPDH (1 : 20000; #5174; cst, USA) overnight at 4°C. After washing the PVDF membrane using TBST 5-6 times, the PVDF membrane was soaked with anti-mouse (1 : 5000; #7076) or anti-rabbit (1 : 5000; #7074) IgG (HRP) secondary antibodies with TBST for 2 h at 37°C. The enhancement solution in the ECL reagent was mixed with the stable peroxidase solution in a ratio of 1 : 1. Then, the mixture was added to the PVDF membrane and protein band was visualized.

### 2.10. Construction of a Gene Signature

Univariate Cox regression analysis was presented for screening survival-related genes with *p* < 0.05. The top 40 genes were selected for multivariate Cox regression analysis with a stepwise method. Finally, a gene signature was constructed. Patients in the training set were separated into the high and low score groups. Kaplan-Meier of overall survival was presented. The prognostic value was validated in the validation set. Furthermore, the predictive independency of this signature was evaluated in different subtypes.

### 2.11. Statistical Analysis

All statistical analyses were conducted using R language (https://www.r-project.org/) and GraphPad Prism 8 (GraphPad Software Inc., La Jolla, CA). *p* value < 0.05 was set as the evaluation criteria.

## 3. Results

### 3.1. Development of Two Distinct Molecular Subtypes for R-CHOP-Treated DLBCL Patients

Totally, 233 R-CHOP-treated DLBCL samples were included in the training set, which were clustered by the ConsensusClusterPlus package in R. When *k* = 2, two molecular subtypes were conducted (Figure 1(a)). Following resampling, the cluster-consensus scores of the two subtypes were both higher than 0.8, indicating that the cluster analysis had high stability (Figure 1(b)). The overall survival results showed that the patients' prognosis was significantly different between the two subtypes (Figure 1(c)). Patients in the subtype I group exhibited a worse prognosis than those in the subtype II group (*p* < 0.0001; Figure 1(c)). This indicated that there was a distinct difference in clinical outcomes between the two subtypes.

RETRACTED

### 3.2. Molecular Subtypes Are Associated with Distinct Clinical Outcomes

Based on the gene expression profiles, feature genes with FDR < 0.05 were screened between subtypes I and II in the training set. According to these feature genes, 383 samples in the validation dataset were divided into two subtypes using the NTP algorithm. As a result, these samples were significantly clustered into subtypes I and II. We further analyzed the differences in overall and progression-free survival time between the two molecular subtypes. The results showed that R-CHOP-treated DLBCL patients in subtype I significantly exhibited shorter overall survival time than those in subtype II (*p* = 0.0041; Figure 2(a)), which were consistent with the results from the training set. Furthermore, we found that patients in subtype I usually experienced poorer progression-free survival time in comparison to those in subtype II (*p* < 0.0001; Figure 2(b)). Also, we performed multivariate Cox regression analysis. Consistently, there were also distinct differences in overall survival and progression-free survival time between the two subtypes after adjusting gene expression profile classifications (Table 2). Thus, the two molecular subtypes could be associated with distinct clinical outcomes.

### 3.3. Different Clinicopathological Features of Molecular Subtypes

We analyzed the differences in clinicopathological features between molecular subtypes via the Wilcoxon rank-sum test. In Figure 3(a), age in subtype I was significantly higher than that in subtype II (*p* < 0.01). Compared to subtype II, there were fewer DLBCL samples at stage 1 in subtype I (*p* < 0.05; Figure 3(b)). In subtype I, more clinical samples were at stage 4 in comparison to subtype II (*p* < 0.01). Thus, these molecular subtypes were highly correlated to the degree of malignancy of DLBCL. As shown in Figure 3(c), there was no statistical difference in sex between the two molecular subtypes (*p* > 0.05). Regarding the international prognostic index (IPI), the percentages of IPI > 3 samples were significantly higher in subtype I than subtype II (*p* < 0.05) in Figure 3(d).

### 3.4. GSEA and Identification of T Cell Exhaustion-Related Genes

To further probe into underlying biological processes of these genes in the two subtypes, GSEA was carried out. Highly expressed genes in subtype I were mainly enriched in lymphocyte activation, T cell activation, regulation of leukocyte activation, cellular response to interferon-gamma, antigen processing and presentation of exogenous peptide antigen via MHC class I, regulation of lymphocyte activation, antigen processing and presentation of peptide antigen via MHC class I, response to lipopolysaccharide, activation of immune response, and lymphocyte proliferation (Figure 4(a)). Highly expressed genes in subtype II were distinctly enriched in extracellular matrix organization, extracellular structure organization, homophilic cell adhesion, cell-cell adhesion, extracellular matrix disassembly, collagen catabolic process, regulation of cellular component movement, regulation of cell migration, regulation of cell motility, and multicellular organismal catabolic process (Figure 4(a)). In Figure 4(b), T cell exhaustion-related genes including TIM3 (*p* < 0.001), PD-L1 (*p* < 0.0001), LAG3 (*p* < 0.0001), CD160 (*p* < 0.001), and CD244 (*p* < 0.001) had distinctly higher expression levels in subtype I than in subtype II.

RETRACTED

### 3.5. Validation of T Cell Exhaustion-Related Genes in DLBCL

qRT-PCR was used to validate the mRNA expression of T cell exhaustion-related genes in 30 paired DLBCL and healthy specimens. Consistent with our bioinformatics results, TIM3 (*p* < 0.001; Figure 5(a)), PD-L1 (*p* < 0.05; Figure 5(b)), LAG3 (*p* < 0.05; Figure 5(c)), CD160 (*p* < 0.05; Figure 5(d)), and CD244 (*p* < 0.05; Figure 5(e)) displayed significantly higher mRNA expression levels in DLBCL than healthy specimens. Consistently, western blot results also showed that TIM3 (*p* < 0.001), PD-L1 (*p* < 0.01), LAG3 (*p* < 0.001), CD160 (*p* < 0.001), and CD244 (*p* < 0.001) proteins exhibited higher expression levels in DLBCL specimens in comparison to healthy specimens (Figures 6(a) and 6(b)).

### 3.6. Development of a Prognostic Gene Signature for DLBCL

By applying univariate Cox regression analysis, 375 survival-related genes were identified for DLBCL. We selected the top 40 genes for multivariate Cox regression analysis. As a result, a 10-gene signature was established, including TRPC4, TIMP1, PPP1R7, NPIPB11, NLK, NCOA1, LMO2, CPNE3, CD3EAP, and CD209 (Figure 7(a)). In the training set, patients with high-risk scores indicated undesirable outcomes than those with low-risk scores (*p* < 0.0001; Figure 7(b)). The predictive efficacy was confirmed in the validation set (*p* < 0.0001; Figure 7(c)). Furthermore, both in the germinal center (GC) and non-GC groups, high-risk scores were indicative of shorter overall and progression-free survival time (Figure 8(a)). For ABC or GCB subtype, high-risk scores predicted poorer survival outcomes (Figure 8(b)).

RETRACTED

## 4. Discussion

R-CHOP can relieve about 60% to 70% of patients. However, the remaining patients may relapse within 2-3 years after treatment [2]. The choice of salvage therapy is very poor, with an adverse reaction rate of about 20%. How to predict the prognosis of patients in the early stage, so as to choose more effective treatment strategies for high-risk patients, is vital to saving lives [2].

Due to the high heterogeneity of DLBCL, it is necessary to identify specific molecular subtypes of DLBCL and identify biomarkers to predict the clinical outcomes of high-risk groups. Herein, DLBCL samples were mainly clustered into the two molecular subtypes (Figures 1(a) and 1(b)). In the training set, patients in subtype I exhibited shorter overall survival time in comparison to those in subtype II (Figure 1(c)). After validation, there were distinct differences in overall survival and progression-free time between the two molecular subtypes (Figures 2(a) and 2(b)). The prevalence of DLBCL in the elderly is increasing [24]. Age over 60 has been considered a risk factor for DLBCL [25]. Increasing age is in association with more complex biological behaviors. Our results showed that patients in subtype I had older age than those in subtype II (Figure 3(a)). Furthermore, compared to the patients in subtype II, more patients are in advanced stages in subtype I (Figure 3(b)). No significant difference in sex was found between the two subtypes (Figure 3(c)). IPI is widely applied for risk stratification of patients with DLBCL (Figure 3(d)). The 3-year overall survival rates of patients with IPI scores of 0-1, 2, 3, and 4-5 were 91%, 81%, 65%, and 59%, respectively [26]. For patients in subtype I, the percentage of IPI score > 3 was distinctly higher than those in subtype II. However, due to the addition of rituximab to the CHOP regimen, the ability of IPI to distinguish high and low risk has decreased. Efforts to characterize the prognosis of DLBCL using immunohistochemistry have identified a variety of genetic markers with prognostic significance. These novel prognostic markers are independent of IPI but have few impacts on their prognostic capacity, largely due to the inherent limitations of the application of these markers [27].

In spite of a deep understanding concerning related signal transduction pathways among high-risk DLBCL populations, randomized phase III trials of integration of targeted therapy and R-CHOP regrettably failed to ameliorate the prognosis of DLBCL patients [28, 29]. 280 highly expressed genes in subtype I were mainly enriched in T cell activation, lymphocyte activation, and immune response (Figure 4(a)). Moreover, cell adhesion, cell migration, and motility were significantly enriched by 585 highly expressed genes in subtype II (Figure 4(a)). In chronic infections and cancer, T cells are exposed to persistent antigens or inflammatory signals. This process is usually related to the deterioration of T cell function. Exhausted T cells lose their effector functions, express a variety of inhibitory receptors, change the expression and use of key transcription factors, develop metabolic disorders, and fail to transition to a quiescent state [30].

RETRACTED

The heterogeneity of clinical outcomes can be partly attributed to genetic heterogeneity [31]. Therefore, we further analyzed the differentially expressed genes between the two subtypes to explain the reasons for the differences in clinical outcomes involving DLBCL patients receiving R-CHOP therapy. Among them, T cell exhaustion-related genes including TIM3, PD-L1, LAG3, CD160, and CD244 were significantly higher in subtype I than in subtype II (Figure 4(b)). TIM3 is a membrane of the T lymphocyte immunoglobulin mucin (TIM) family, which is expressed in T helper 1 (Th1) and cytotoxic T cells (Tc1). As a negative regulator, it induces the apoptosis of Th1 and Tc1 cells [32]. Compared with healthy controls, DLBCL patients have higher expression of TIM3. Its expression was positively related to the DLBCL stage [33]. TIM3 expression can reflect the treatment efficiency of patients with chemotherapy [33]. LAG3 is a member of the immunoglobulin superfamily, which acts as a negative regulator of T cell homeostasis [34]. LAG3 is coexpressed with TIM3 and PD-L1 in DLBCL [34]. CD160 is an Ig-like glycoprotein expressed by natural killer cells and T cell subset [35]. Upregulation of PD-L1 can increase the immune escape of cancer cells in DLBCL [36]. CD244 is a family member of the signal lymphocyte activation molecule of immune cell receptors [37]. Our qRT-PCR and western blot confirmed the higher expression of TIM3, PD-L1, LAG3, CD160, and CD244 in DLBCL (Figures 5 and 6). Finally, we developed a 10-gene signature for predicting the prognosis of DLBCL patients (Figures 7 and 8). Thus, our research might provide potential information for precise drug treatment strategies and prognosis prediction for DLBCL.

Taken together, we constructed and confirmed two molecular subtypes of DLBCL with distinct prognosis features. The molecular subtype classifications may be adapted to the real world. In our future studies, we will validate the classifications in our DLBCL cohort. Moreover, several feature genes were identified, which might become promising therapeutic targets for future immunotherapy. Despite these feature genes being validated via qRT-PCR and western blot, their functions should be verified in a larger cohort of DLBCL.

RETRACTED

## 5. Conclusion

In this study, we constructed and externally verified two novel molecular subtypes with distinct prognosis and clinical characteristics for DLBCL by consensus cluster analysis, which could be used for risk stratification and prognosis prediction in clinical practice.

## Figures and Tables

**Figure 1:** Development of two distinct molecular subtypes for R-CHOP-treated DLBCL patients. (a) A consensus matrix heat map when *k* = 2. The row and column of the matrix represent different samples. The values of the consensus matrix range from 0 (cannot be clustered together) to 1 (always clustered together) in white to dark blue. The consensus matrix is arranged in accordance with the consistency classification (the tree diagram above the heat map). (b) Cluster-consensus scores of the two molecular subtypes when *k* = 2. The higher the score, the higher the stability. (c) Kaplan-Meier overall survival analysis for patients in the two molecular subtypes. Red represents the subtype I group, and blue represents the subtype II group.

**Figure 2:** Molecular subtypes are associated with distinct clinical outcomes. (a) Overall survival analysis of R-CHOP-treated DLBCL patients in subtypes I and II. (b) Progression-free survival analysis of patients in subtypes I and II. Red represents subtype I, and blue indicates subtype II.

**Figure 3:** Correlation between different clinicopathological features and molecular subtypes. (a) Violin diagram depicting the differences in age between the two molecular subtypes. (b) Stage distributions between the two molecular subtypes. (c) Sex distributions of samples between the two molecular subtypes. (d) Differences in international prognostic index (IPI) between the two molecular subtypes. NS: *p* > 0.05; ^∗^*p* < 0.05; ^∗∗^*p* < 0.01.

**Figure 4:** GSEA and identification of T cell exhaustion-related genes. (a) The top ten biological processes enriched by highly expressed genes in subtype I or II, respectively. Blue bubbles represent the annotation results of highly expressed genes in subtype I. Red bubbles express the annotation results of highly expressed genes in subtype II. The size of the bubble is proportional to the number of enriched genes. The darker the color, the smaller the adjusted *p* value. (b) Violin diagram showing the expression of T cell exhaustion-related genes including TIM3, PD-L1, LAG3, CD160, and CD244 between subtypes I (red) and II (blue). ^∗∗∗^*p* < 0.001; ^∗∗∗∗^*p* < 0.0001.

RETRACTED

**Figure 5:** Validation of T cell exhaustion-related genes in DLBCL via qRT-PCR. The mRNA expression levels of TIM3 (a), PD-L1 (b), LAG3 (c), CD160 (d), and CD244 (e) were compared between DLBCL and control specimens. ^∗^*p* < 0.05; ^∗∗∗^*p* < 0.001.

**Figure 6:** Western blot detecting the expression of T cell exhaustion-related genes in DLBCL. (a) Representative images of western blot results. (b) The protein expression levels of TIM3, PD-L1, LAG3, CD160, and CD244 were compared between DLBCL and control specimens. ^∗∗^*p* < 0.01; ^∗∗∗^*p* < 0.001.

**Figure 7:** Establishment and validation of a 10-gene signature for DLBCL. (a) Forest plot for the hazard ratio of the 10 genes in this signature. (b, c) Kaplan-Meier curves of overall survival in the (b) training and (c) validation sets.

**Figure 8:** Subgroup survival analysis of the 10-gene signature for DLBCL. (a, b) Kaplan-Meier curves of overall and progression-free survival in the (a) GC and non-GC groups as well as (b) ABC and GCB subtypes.

**Table 1:** Primer sequences for quantitative real-time PCR.

Target	Primer sequence (5′-3′)	Product (bp)
h-GAPDH-F	ACAACTTTGGTATCGTGGAAGG	101
h-GAPDH-R	GCCATCACGCCACAGTTTC	

h-TIM3-F	TTGGACATCCAGATACTGGCT	86
h-TIM3-R	CACTGTCTGCTAGAGTCACATTC	

h-PDL1-F	TGGCATTTGCTGAACGCATTT	120
h-PDL1-R	TGCAGCCAGGTCTAATTGTTTT	

h-LAG3-F	GCCTCCGACTGGGTCATTTT	131
h-LAG3-R	CTTTCCGCTAAGTGGTGATGG	

h-CD160-F	GCTGAGGGGTTTGTAGTGTTT	154
h-CD160-R	GTGTGACTTGGCTTATGGTGA	

h-CD244-F	TCGTGATTCTAAGCGCACTGT	237
h-CD244-R	CAGGTTCTTGTGACGTGGGAG	

**Table 2:** Independence of the two subtypes in overall and progression-free survival prediction.

Survival	Variables	coef	exp(coef)	se(coef)	*z*	*p*
Overall survival	Group: II	-1.1084	0.3301	0.3426	-3.2348	6.09*E* − 04
	Subtype: GCB	-0.7356	0.4792	0.3571	-2.0599	3.94*E* − 02
	Subtype: UC	-0.6358	0.5295	0.4019	-1.5820	1.14*E* − 01

Progression-free survival	Group: II	-1.3205	0.2670	0.3258	-4.0535	2.52*E* − 05
	Subtype: GCB	-0.4108	0.6631	0.3380	-1.2154	2.24*E* − 01
	Subtype: UC	-0.4443	0.6412	0.3687	-1.2053	2.28*E* − 01

Abbreviations: coef: coefficients; exp: exponential; se: standard error; *z*: *z*-score; *p*: *p* value; GCB: germinal center B cell; UC: unclassified.

## Data Availability

The datasets analyzed during the current study are available from the corresponding author on reasonable request.

## Abbreviations

DLBCL: Diffuse large B cell lymphoma
GSEA: Gene set enrichment analysis
IPI: International prognostic index
R-CHOP: Rituximab, cyclophosphamide, doxorubicin, and prednisone
GEO: Gene Expression Omnibus
FDR: False discovery rate
NTP: Nearest template prediction
GO: Gene Ontology
qRT-PCR: Quantitative real-time PCR
coef: Coefficients
exp: Exponential
se: Standard error
*z*: *z*-score
*p*: *p* value
GCB: Germinal center B cell
UC: Unclassified.
